The article "Influence of Diversified Health Elements Based on Machine Learning Technology on Pop Vocal Singing in a Cultural Fusion Environment" was retracted in 2023. Reasons: unreliable results or conclusions; concerns about the data; concerns about the results or conclusions; concerns about the peer review.

# Influence of Diversified Health Elements Based on Machine Learning Technology on Pop Vocal Singing in a Cultural Fusion Environment

**DOI:** 10.1155/2022/7903838

**Published:** 2022-09-26

**Authors:** Han Xia

**Affiliations:** Shenyang Conservatory of Music, Modern Conservatory of Music, Department of Popular Vocal Music, Shenyang, Liaoning Province 110168, China

## Abstract

The multicultural environment is affected by the ongoing advancement of science and technology, which results in more and more planned cultural fusions and collisions between various cultures. The emergence of distinct national cultures has emphasised cultural diversity. Music naturally takes the initiative and promotes diversity in social and cultural awareness as a cultural art form with distinctive charm. Cultural variables play a significant role in the development, appeal, and wide transmission of voice output. It is an authentic catharsis and a vivid record of spiritual activity among people. Because the diversity of art is also the source of the legacy and growth of creative innovation, the diversified integration of art will also promote the shared development of all nations. Vocal music and singing art must adapt to the circumstances, follow the trend of the times, and grow slowly and healthily in the direction of diversity in the context of multicultural development. Musical emotion is the key component of music. The periodic properties of sound should be studied since they have important implications for music study. In order to learn and predict the 8-dimensional emotion vector of musical compositions, this study creates a dataset of 200 pieces of music, isolates music emotion detection as a regression issue, and applies machine learning techniques. According to experimental findings, when mid- and high-level characteristics are used as input instead of low-level features, accuracy can increase from 50.28% to 68.39%.

## 1. Introduction

In the process of singing, music can express its content and emotions through popular language for people to enjoy. Pop music is one of many forms of music. Pop music is full of vitality and artistic charm. It is often sung in different forms and is deeply loved by people [1]. In the process of singing popular music, singers can express the music in different forms through their own understanding of vocal music, so that people can understand popular music from various angles. The development of music is closely related to the development of contemporary society. As a part of music art, singing art form is indispensable [2]. The progress of society, the development of productive forces, and the exchange of culture have all promoted the development of vocal singing forms in music art towards diversification [3]. In the high-tech era, the speed of music transmission is fast, the public has a wide range of ways to obtain music, and their musical literacy is getting higher and higher. Therefore, when the public is used to listening to excellent music works from all over the world, the single vocal singing form can no longer be satisfied by the public, and even audio-visual “fatigue” will appear [4]. In this situation, the integration of new singing forms is a necessary way to satisfy the appreciation of popular music for the discovery of new things, and then, the so-called “cross-border music” appeared, which is the most diversified development of pop music [5].

Music in the twenty-first century is a multicultural art value, and then, the visual art of popular vocal music should also create some concepts in the music world. Blues and ragtime, jazz, blues, rhythm, big band swing, country music, popular vocal music, and now popular connection has established many elements. We see a pop vocal art [6]. As an important performing art, pop vocal music has different values and aesthetic forms. Theme in different periods, work style, and singing have different connotations and meanings, and of course, they can also produce different musical and artistic effects [7]. Pop vocal singing, in fact, is very common, simple imitation, or interpretation of deep thoughts in every work content and art. Everyone must fully understand the creation of the artistic style of singing. The structure of the creation work itself is very simple. Effective and pleasant melodies, analysis, and understanding are a kind of ability to promote the ability and expand the aesthetic field [8]. However, music's main component is music emotion, and research on music information behaviour shows that people frequently utilise emotion as a criterion for retrieving music. The nerve system only responds positively to periodic sounds, according to the human auditory system, and uncomfortably to nonperiodic impulses. As a result, learning about the periodic properties of sound is useful for studying music. In order to increase the accuracy of automatic music emotion detection from a feature perspective, this study primarily examines the impact of middle, high, and low-level features as model input on the performance of the music emotion recognition model.

From the perspective of cultural integration, vocal performances are constantly developing in a diversified direction. First of all, people accept and recognize the scientificity and rationality of the bel canto, which is the focus of concept fusion and theoretical research. Secondly, comprehensively analyze and summarize the characteristics of their own development and identify areas that need to be improved. Finally, after comparing the artistic characteristics of Chinese and Western vocal music, we will find a suitable point for integration and development in the relevant aspects of creation, singing, and performance. In terms of communication methods, compared with traditional communication channels such as radio and television, the Internet and mobile phones have the advantages of being faster and more convenient [9]. New media audiences such as Tiktok, WeChat, online live broadcast, and video platforms are more extensive. People's appreciation of vocal music art is no longer limited by time and space which greatly promotes the communication and dissemination of modern vocal music performance at home and abroad and fully shows the excellent traditional culture to the world.

Under such a background, many ethnic elements have been expressed with more modern characteristics in the integration. The cultures and even languages of many ethnic groups have become popular in the world. This will strengthen the confidence of our nation in developing its own culture, enhance the depth and recognition of our culture, and make us more confident [10]. The significance of this study lies in the following: (1) the classification of songs with different emotions can be realized using chord recognition technology. Because the same chord sequence often expresses similar or even the same music style or emotion, the more the repeated parts of the chord segments of two pieces of music, the higher the similarity of the two pieces of music, or the more similar the music emotion expressed. (2) At the same time of spectrum energy compression, the harmonic information is mapped by the normalization method. This method can not only effectively weaken the influence of the instrument category on the chord characteristics but also reduce the influence of the singer's timbre.

This article is organized into seven sections: the first section is the introduction part. This part analyzes that under the background of multicultural development, vocal singing art, as the main art form, must keep pace with the times, keep up with the trend of the times, and develop steadily and healthily in the direction of diversification. Studying the periodic characteristics of sound is instructive for studying music. The second section mainly summarizes the relevant literature, summarizes the advantages and disadvantages, and proposes the research ideas of this paper. The third section introduces vocal art and music and singing feature extraction in detail. In the fourth section, the algorithm analysis is carried out with the dataset of 200 music clips as samples. The fifth section is the experiment and results. The sixth section looks forward to the strategies for the diversified development of popular vocal music. The seventh section concludes, summarizing the findings of the full text.

## 2. Related Work

Ji-Jun believes that with the continuous development of art forms over the past decades, Bel Canto and pop and Bel Canto and national singing are organically combined and integrated. How to absorb the essence of foreign culture while safeguarding the unique characteristics of vocal music art has become a topic that we need to discuss together [11]. Yang emphasized that vocal music culture is the most flexible form of mass culture and art performance. Individuals or people can participate in music and cultural activities anytime and anywhere, without complex environment or facilities, and without a large number of venues [12]. Deng believes that vocal music singing does not only mean how consummate the singing technique is, how good the singing method is, and how deep the works are handled but also that the singing should be closer to the masses and the people during the singing process [13]. Based on such a cultural integration perspective, vocal music art, as the carrier of culture, naturally has been more rapidly and fully integrated, playing the effect of cultivating the humanistic spirit. Wang et al. elaborated and explored the effect of vocal music art on the cultivation of urban humanistic spirit to achieve the purpose of practical application [14]. Cahn pointed out that the main feature of vocal music art based on cultural integration is cultural integration. Only through sustained and effective communication on multiple platforms can we continuously promote the development of vocal music art, thus completing the cultivation of urban humanistic spirit [15]. Klement and Strambach research points out that popular music is spreading widely, and this recognized beauty of music is not pure objectivity, which reflects a strong subjectivity of the public's aesthetics. For music, a magical culture, it is emotional and casual [16]. Investigate and examine the issues with polyphony estimate and melody extraction in music. People's sense of musical rhythm is largely dependent on the periodicity of the signal energy's strength, allowing for frequency domain analysis of the energy signal. The bridge connecting music applications and actual music is music recognition technology. In light of this, Oliveira et al. invited 60 musicians to express various emotions such as joy, sorrow, fear, and calm by manipulating the numerical combination of 7 characteristic quantities such as rhythm and timbre in the device, and he then discovered a relationship between these characteristics and musical emotions [17]. Wei et al. develop a recommendation model that is based on musical emotion and primarily examine the emotion that movie music conveys [18]. To anticipate the emotional worth of music and to identify its emotional content, Lin and Wang employ a continuous emotional mental model, regression modelling, and two fuzzy classifiers that evaluate emotional intensity [19]. Yan proposed the Mel tone contour feature after integrating the pertinent knowledge of music theory with the auditory characteristics of the human ear. The typical tone contour feature's tendency to blur when the frequency is low is remedied by this chord feature [20].

## 3. Vocal Music Art and Singing Feature Extraction

Music is an important means that people gradually explore to express their emotions in the process of life. Music art has the characteristics of wide spread and strong appeal, which can not only cultivate the artistic sentiment of the people but also enrich the amateur life of the people and promote the harmonious development of community civilization. Through music training, make the mass cultural activities more colorful [21]. People sing according to their emotions, sometimes giving out single tones of different intensities and pitches. Sometimes, in order to express more complex emotions, it is necessary to generate specific resonance by superimposing multiple sounds according to a certain relationship. From another perspective, people or machines can also extract some specific features from the singing music, such as chord, pitch, tonality, etc., to grasp the specific emotions to be expressed in the music. Therefore, the music contains a lot of hidden information that the music player wants to express. If we want to deeply understand a piece of music, we need to deeply study the high-level features contained in the music.

The fundamental principle of vocal singing fluency is to maintain the highest note while omitting lower-pitched tones (as shown in Figure 1). The main melody's pitch is often higher than the accompaniment melody's in most compositions. For the majority of musical compositions, the fundamental contour method is appropriate; nevertheless, the pitch feature cannot be employed as a criterion for evaluating the main melody in a few compositions with high accompaniment melody.

Most popular songs are a mixture of singing and accompaniment, while many music applications, such as theme extraction, singer recognition, and lyrics recognition and alignment, are only related to the singing. From the perspective of music theory and music expression, the music features of the three levels can be described as basic features, partial features, and overall features (see Figure 2). Because the original audio signal hardly contains any high-level music features such as music emotion and music genre. If the feature can express the content of the whole music, such as music style and music emotion, then this feature is called the overall feature, also called the high-level feature. Therefore, most audio-related application systems are related to audio frequency domain information. The time-frequency conversion stage of audio signal becomes the most important stage of the whole audio-related application.

Based on the emotional model, this paper uses an 8-dimensional vector to represent the emotional features expressed in a singing segment, in which 8 dimensions, respectively, represent 8 emotional sets in the emotional model: holiness, sadness, yearning, lyricism, lightness, happiness, enthusiasm, and vitality. The numerical value of each dimension in the emotion vector reflects the intensity of the emotion in the segment. The model proposed in this paper abstracts music emotion recognition as a regression problem and uses machine learning method to learn manually labeled samples and their features and obtains a prediction model, so that the emotion vector of music segments can be automatically predicted by inputting the features of music segments, as shown in Table 1.

As digital technology has advanced quickly, it has become popular to create music databases using music formats that are very adaptable. Sound files are binary data that have been converted from samples of actual sound waveforms. Sampling frequency, depth, and environment have a significant impact on the quality of sound files, meaning that different data may be collected for the same sound.

## 4. Algorithm Analysis

A total of 100 volunteers were requested to evaluate the music snippets subjectively during the entire experiment. In order to ensure that each sample segment was annotated by at least 10 distinct volunteers, each volunteer was asked to annotate 36 randomly chosen music parts. 64 soundtrack songs with complete scores were chosen from a total of 100 soundtrack songs that were pulled from the current popular vocal music tracks. They were intercepted into 928 29-second segments, and 450 useful portions were chosen at random to serve as the sample segments for labelling in this experiment. Choose 70 complete soundtracks, divide them into 200 segments of 20 seconds each, and then, pick 150 of the 200 segments at random to serve as the test segments for this experiment's labelling. Finally, a dataset of 200 music clips is created, and music emotion recognition is abstracted as a regression issue. The period component of the energy signal is determined in the whole song, this period is also the rhythm of music singing, and its formula is expressed as:

(1) $$\begin{array}{c} E_{n}=\overset{\infty }{\underset{m=-\infty }{\sum }}x{\left(m\right)}^{2}. \end{array}$$

Nonlinear fitting is carried out in the multidimensional space, and the numerical relationship between the features will not affect the final learning result. It is only necessary to ensure that the values corresponding to different situations under the same feature are unique and fixed.

(2) $$\begin{array}{c} \theta =\frac{1}{N}\overset{n}{\underset{i=1}{\sum }}\left(y_{i}-r{\left(x_{i}\right)}^{2}\right., \end{array}$$

where *x*_*i*_ is the feature vector of the *i*th input singing segment and *y*_*i*_ is the actual emotional value of the singing segment, that is, the predicted target.

Each track channel has a sound image adjustment value pan, which is used to indicate the position of the sound source, and the range is 0-102. When pan = 54, the sound source is balanced. If pan is too large or too small, the sound source is unbalanced. The balance degree of the music sound source is represented by the feature quantity *F*_0_:

(3) $$\begin{array}{c} F_{0j}=1-\frac{\left|{\text{Pan}}_{j}-48\right|}{127}. \end{array}$$

Among them, *j* is the track symbol, and *j* = 1, 2, ⋯, 126.

Pitch refers to the high or low frequency of a note, expressed in pitch. The pitch feature can be directly extracted from the melody of the singing music, and the range is 0-98. On the basis of extracting the melody of a certain track channel, the average pitch of a certain track channel can be obtained by calculating the average pitch of the melody notes, which is defined as the feature quantity *F*_1_.

(4) $$\begin{array}{c} F_{1j}=\frac{1}{n}\overset{n}{\underset{i=1}{\sum }}{\text{pitch}}_{1j}, \end{array}$$

where *n* is the number of notes of track *j* and pitch_1*j*_ is the pitch of the first note in the melody of track *j*.

According to the extracted features, the track channel where the main melody is located can basically be determined. The judgment result is expressed as function *Y*(*k*), that is, the score that the *j*th track channel in the music file contains the main melody, as shown in

(5) $$\begin{array}{c} Y\left(k\right)=\frac{1}{4}\overset{4}{\underset{m=1}{\sum }}a_{m}{F_{jm}}^{2}. \end{array}$$

Among them, *j* = 1, 2, 3, 4.

From this, the feature score table of the audio track of the music piece is obtained, as shown in Table 2.

In addition to these parameters, for the case where the target information is human voice, the voice recognition technology and musical instrument classification technology can also be used to judge whether there is sound or not. If the human voice is regarded as a special musical instrument, many features applied to the classification of musical instruments can also play a role in the judgment of voiced and voiceless. In speech recognition, there is also the problem of human voice segment recognition. Based on the similarity of human voices in speech and music, it is also reasonable to borrow speech recognition technology. Short-time Fourier change is introduced, and a small segment of the signal is taken out of the signal with a window function of appropriate width for Fourier transform, to obtain the local spectrum during this time. The short-time Fourier transform is defined as follows:

(6) $$\begin{array}{c} X\left(w,t\right)=\int_{-\infty }^{\infty }x\left(t\right)*w\left(\lambda -\eta \right)*e^{-wt}d\eta . \end{array}$$

In the formula, *x*(*t*) is the time signal, *w*, *t* is the window signal, and *X*(*w*, *t*) is the spectrum at the time of *t*.

By definition, we know that time-stretching of music only changes the length of time (i.e., the speed) of the music signal and not the pitch. Therefore, after time stretching, the spectrogram image of the music signal should remain stable on the frequency axis, but only the time axis is stretched or shortened.

(7) $$\begin{array}{c} y\left(f\right)=\left[1.2\times \log_{2}\frac{f}{f_{0}+f_{1}}+1\right]. \end{array}$$

Note that the positional change of the energy of the signal component on the frequency axis is independent of the value of *f*, as shown in the following formula:

(8) $$\begin{array}{c} y\left(\left(i+k\right)f-y\left(f\right)\right)=\left[1.2\times \log_{2}\left(1+k\right)\right]. \end{array}$$

In the real-world songs, melody is the most prominent one at present. It has the largest energy and is most easily recognized. In the task of melody extraction, we should make full use of its own characteristics. According to the previous introduction of various sound and no sound judgment parameters, energy is finally selected as the sound and no sound judgment parameter. Here, we will compare the two energy expressions, energy and logarithmic energy, and define them as follows:

Energy:

(9) $$\begin{array}{c} E=\sum s^{2}\left(n\right). \end{array}$$

In the formula, *E* represents the energy of a certain frame, and *s*(*n*) is the sampled value of point *n*.

Logarithmic energy:

(10) $$\begin{array}{c} E_{s}=50\text{dB}+10\log_{2}\left(\sum s^{2}\left(n\right)\right), \end{array}$$

where *E*(s) represents the logarithmic energy of a frame and 50 DB is added to the expression to ensure that the final result is positive.

Different thresholds will be set to determine the beginning and ending points of the spoken segment based on the features of high intensity at the beginning and low intensity at the conclusion of the sound. The music is not preprocessed using techniques like filtering before deciding if there is sound or not. This is because we want to give the melody extraction process as much spectrum data as we can. Although the range of human voice pitch is limited, harmonics have no such restrictions. In order to preserve as much of the input music's spectrum information as possible, it is not preprocessed. The output frequency is reduced when the final pitch sequence is output to eliminate frequencies that are unlikely to be heard in singing.

## 5. Experiments

Before emotion recognition, emotion-related features need to be used as the input of the recognition model, and emotion feature analysis is the basis for the accurate establishment of emotion recognition models. When extracting the emotional features of music, the most used ones are the low-level features of music, such as MFCC, LPC cepstrum, zero-crossing rate, short-term energy, spectral centroid, and other features. However, the correct rate of identifying high-level emotions through low-level features is not high. The characteristics that affect the emotional calculation of music mainly include mode, speed of sound, rhythm, beat, pitch, sound intensity, and melody.

From the amplitude of the music waveform segment selected in Figure 3, it can be seen that when the current state is silent, only when the energy of this frame is greater than the threshold value will it be judged that the *θ*_1_ break is called sound. When the current state is sound, only when the energy of this frame weakens to less than the threshold value *θ*_2_ will it be judged as no sound. The frame judged as having sound will continue to perform the subsequent stage, and the frame judged as having no sound will be terminated, and the frequency *F*_0_ = 0Hz will be output. In the experiment, the judgment results of different energy expression methods will be compared, and the more effective way will be selected as the final use through the comparison results.

First, the real-time singing signal is input through the microphone and stored in wave format. Then, the melody of the singing signal is extracted through the new algorithm in this chapter and compared with the standard melody to determine whether the singing is accurate. Finally, both the singer's melody curve and the standard melody curve are displayed on the system interface in real time to help users visually observe their performance. It can be seen from Figure 4 that the reason why the accuracy rate is improved when the middle and high-level features are adopted is that compared with the low-level features, the middle and high-level features have stronger and more direct correlation with emotion. From the perspective of musical theory, the value of each middle and high-level feature can often clearly reflect the emotional trend of a piece of music.

It can be seen from Figure 5 that, judging from the importance of the model output, the order of contribution rate of each feature to the accuracy of music emotion recognition is: speed > mode > melody trend > musical instrument > chord > texture > beat. After the signal is sampled and quantized, the amount of data is usually relatively large, and the frequency of music rhythm is relatively low. In the analysis, only low-frequency components are concerned. In order to save the operation cost, the signal is extracted by integer multiples.

Unlike iterative estimation methods, joint estimation methods simultaneously evaluate the likelihood of a set of fundamental frequencies, rather than considering each fundamental frequency individually. Although an iterative extraction and suppression process is not required, coincident harmonics are still a problem in joint estimation. Some methods obtain a multitone confidence function by combining the confidence functions of several single-tone estimates to evaluate the likelihood of a set of fundamental frequencies.

The competitiveness of our singing voice separation algorithm decreases as the singing voice to music ratio increases. The more energetic the vocals, the more difficult it is to model and reduce the instrumental sounds, and thus the less well separated our vocals are. At the same time, musical chords do not exist in isolation, and this feature is inextricably linked with other features of music. Combining other features of music to generate joint chord features will also greatly improve chord recognition. Unlike speech, music has a more complex spectrum structure (as shown in Figure 6). In addition, the music signal is easily interfered by the external environment, so that the research materials obtained by researchers are not very ideal. This requires researchers to combine with deep knowledge of music theory and start from music theory, to dig out characteristic quantities that can more powerfully express the characteristics of signal chords.

In the face of a variety of music in real life, we need to use a more fault-tolerant method, such as limiting the frequency range for harmonic matching. According to the above steps, if the song sung is “song a,” according to Figure 7, the peak position in the normalized digital frequency ar map is at point 29, and the corresponding frequency is 1.24 hz, which is the stress beat cycle of the song There are also several spectral peaks in Figure 7, which are 55 points and 84 points, respectively, and the corresponding frequencies are 2.36 hz and 3.61 hz. These frequencies are harmonic components of the accent frequency.

The high-level features such as speed, beat, texture, rhythm type, melody trend, mode, and chord are manually marked out from the music, and the modeling is carried out using machine learning algorithm. The experimental results show that the recognition accuracy of the model is significantly improved when the middle- and high-level features are used as the input, compared with the low-level features. Compared with the low-level features, the accuracy rate can be improved from 50.28% to 68.39%. Accurate estimation of the location of harmonics in recorded audio can obtain good results, but for synthetic audio without harmonic offset, this method becomes inappropriate.

## 6. Diversified Development Strategy of Pop Vocal Singing

With the surging tide of the times, the unremitting pursuit of human survival ideals and aesthetics, and the pace of the development of spiritual civilization in contemporary society, the accumulation and definition of vocal music has entered a full and brand-new historical stage. The interaction between music creation and singing art has a very clear expression in various singing methods such as “Bel Canto,” “national,” and “popular.” The fusion and innovation of the diversified styles of song creation have been fully demonstrated on the stage through the wonderful deduction of singers and stars. It is necessary to establish a correct concept of vocal music, break the traditional concept and the concept of division of singing methods, hold the idea of respect, absorption and innovation, and form a diversified vocal music cultural mind and an aesthetic concept in which various singing methods can coexist. Therefore, we should develop diversified vocal singing art from many aspects.

1. Increase cultural identity among ethnic groups and promote cultural communication and integration among ethnic groups. Whether it is economic or cultural, diversified development has become the mainstream of social development. Therefore, we should follow the trend, integrate the current elements into the national vocal music, and learn from the advanced skills of other nationalities to improve the artistry of the national vocal music art and better meet the requirements of the people for vocal music art
2. Provide a multidimensional platform for vocal art exchange. With the help of current scientific and technological means, we will launch more platforms for vocal music art exchange, create a vocal music art exchange system with urban characteristics, and let more grass-roots personnel participate in it to acquire knowledge of vocal music art. For example, we can try to hold relevant competitions and use the publicity media of WeChat platform to expand the influence of vocal music art and promote the cultivation of humanistic spirit
3. Strengthen the input of the related foundation of vocal music art. Increase the city's relevant foundation's intake of vocal music art. To promote and cultivate the fundamental vocal music art, it is essential that local culture be fully taken into account from design to construction. It is best to identify the historical and modern characteristics of the city's unique vocal music art. Invest more in fundamental vocal music education, create community-based exhibition and training spaces for vocal music art, and gradually instill a love of vocal music in the hearts of the populace in order to cultivate a humanistic attitude

## 7. Conclusion

The art of modern pop vocal singing is an important manifestation of the development of national culture. Under the background of cultural integration, the development of vocal singing shows diversity, and its musical form, artistic features, singing methods, and musical styles all reflect the trend of diversity and integration. Cultural integration can effectively promote cultural exchanges and the cultivation of humanistic spirit. In today's urban cultural construction, it is necessary to give full play to the unique role of vocal music and get out of the predicament and trap of humanistic spirit cultivation, so as to effectively explore the road of simultaneous development of humanistic spirit in the current economic development and constantly explore the way of humanistic spirit cultivation with urban characteristics. The role played by vocal music and its bearing capacity as a carrier should be fully recognized, and the development path should be found through continuous practice and exploration. The organic combination of Chinese and foreign vocal music culture and the organic combination of national style and local color have played a huge role in identifying the direction and pointing the way to the continuous development of modern popular vocal music, and it is also a special artistic insight with foresight, professionalism, and science.

## Figures and Tables

**Figure 1:** Melody recognition process in vocal singing.

**Figure 2:** Classification of music features.

**Figure 3:** Amplitude of a music waveform segment.

**Figure 4:** Comparison of main scale time-domain variance of different smoothing methods.

**Figure 5:** Accuracy of different emotion categories when entering the model.

**Figure 6:** Multitone estimation results of audio files with different numbers of notes.

**Figure 7:** Importance ratio of singing features.

**Table 1:** Sound features extracted by audio analysis software.

Extraction means	Characteristic dimension	Feature description
PsSound	29	Loudness, sharpness, sound pressure
Msroyas	4 U	Spectral characteristics
General comparison	49	Subband peak, subband valley
DKOP	39	Wavelet coefficient

**Table 2:** Standardized data of music singing characteristics.

Serial number	Average treble	Average intensity of sound	Pitch stability	Sound intensity stability	Speed	Melody direction
1	0.160	-0.004	-0.041	-0.064	0.186	0.295
2	-0.013	0.196	0.286	0.228	-0.012	0.218
3	0.293	0.205	-0.027	0.234	-0.011	0.135
4	0.135	0.087	-0.073	0.191	-0.066	0.155
5	0.062	-0.028	0.000	0.284	0.049	0.394
6	0.194	-0.061	-0.093	-0.022	0.141	0.319
7	0.148	0.261	0.158	-0.069	0.246	0.121
8	0.058	0.074	0.226	-0.007	-0.063	0.249

## Data Availability

The data used to support the findings of this study are available from the corresponding author upon request.
